# HnRNP A1 - mediated alternative splicing of CCDC50 contributes to cancer progression of clear cell renal cell carcinoma via ZNF395

**DOI:** 10.1186/s13046-020-01606-x

**Published:** 2020-06-19

**Authors:** Guoliang Sun, Hui Zhou, Ke Chen, Jin Zeng, Yangjun Zhang, Libin Yan, Weimin Yao, Junhui Hu, Tao Wang, Jinchun Xing, Kefeng Xiao, Lily Wu, Zhangqun Ye, Hua Xu

**Affiliations:** 1 Department of Urology, Tongji Hospital, Tongji Medical College, Huazhong University of Science and Technology, Wuhan, 430030 P.R. China; 2 Hubei Institute of Urology, Wuhan, 430030 P.R. China; 3 Department of Molecular and Medical Pharmacology, David Geffen School of Medicine, University of California at Los Angeles, Los Angeles, CA 90095 USA; 4 Department of Urology, The First Affiliated Hospital of Xiamen University, Xiamen, 361000 P.R. China; 5 Department of Urology, The People’s Hospital of Shenzhen City, Shenzhen, 518000 P.R. China

**Keywords:** ccRCC, CCDC50, Alternative splicing, HnRNP A1, ZNF395

## Abstract

**Background:**

Aberrant alternative splicing events play critical roles in carcinogenesis and progression of many cancers, while sparse studies regarding to alternative splicing are available for clear cell renal cell carcinoma (ccRCC). We identified that alternative splicing of coiled-coil domain containing 50 (CCDC50) was dysregulated in ccRCC, whereas the clinical significance of this splicing event and its splicing regulation mechanisms were still elusive.

**Methods:**

Bioinformatic algorithm was utilized to identify significant exon skipping events in ccRCC via exon sequencing data from The Cancer Genome Atlas. Semi-quantitative real-time polymerase chain reaction and western blot were used to validate the aberrant expression of different transcripts in renal cancer tissues, cell lines and corresponding noncancerous controls. Short hairpin RNA targeting CCDC50 and overexpressing plasmids for each transcript were introduced into ccRCC cell lines, followed by a series of in vitro and in vivo functional experiments. Moreover, a panel of splicing factors were identified and their roles on splicing regulation of CCDC50 precursor mRNA (pre-mRNA) were studied. Furthermore, RNAseq data were analyzed to elucidate downstream molecules of CCDC50. Two-way analysis of variance and unpaired Student t test were used in statistical analysis.

**Results:**

Pre-mRNA of CCDC50 generated two transcripts, full-length transcript (CCDC50-FL) and truncated transcript (CCDC50-S) with exon 6 skipped. CCDC50-S was overexpressed in ccRCC tissues and cell lines compared to noncancerous counterparts, but CCDC50-FL was only detected in noncancerous tissues and normal renal epithelial cells. Higher percent spliced-in index was associated with better survival in ccRCC patients. In vitro and in vivo functional experiments indicated that CCDC50-S transcript promoted the proliferation, migration, invasion and tumorigenesis of ccRCC, while CCDC50-FL exerted opposite tumor suppressive functions. Besides, we identified that heterogeneous nuclear ribonucleoprotein A1 (HnRNP A1) could promote the skipping of exon 6, which resulted in higher portion of CCDC50-S and oncogenic transformation. Moreover, zinc finger protein 395 (ZNF395) was identified as a downstream protein of CCDC50-S, and the interaction initiated oncogenic pathways which were involved in ccRCC progression.

**Conclusions:**

Aberrant alternative splicing of CCDC50 is regulated by HnRNP A1 in ccRCC. This splicing event contributes to cancer progression through the downstream pathway involving ZNF395.

## Background

Renal cell carcinoma (RCC) represents a group of histologically and molecularly heterogeneous cancers which are originated from renal epithelium. Approximately 295,000 newly-diagnosed cases and 134,000 deaths of RCC are documented annually worldwide [1]. The most common subtype of RCC is clear cell renal cell carcinoma (ccRCC), which is the main culprit for majority of cancer-related deaths. Previous studies have identified the somatic von Hippel-Lindau (VHL) mutations and downstream hypoxia-inducible factors (HIFs) - related pathways in the carcinogenesis of ccRCC, while recent high-throughput sequencing also identifies aberrant changes in epigenetic regulatory genes or precursor mRNA (pre-mRNA) splicing [2]. Besides, extensive studies have revealed the remarkable genetic diversity in ccRCC, which shed light on the correlation between these molecular events and aggressive clinical features in ccRCC and exhibit prognostic, predictive and therapeutic relevance [3]. Given that metastatic ccRCC is not suitable for surgery and refractory to conventional radiotherapy and chemotherapy, potential future directions for ccRCC management should be based on thorough investigations in ccRCC pathophysiology, which is promising for providing novel molecular targeted agents and reliable biomarkers.

Alternative splicing is a post-transcriptional regulatory mechanism of gene expression which modulates distinct protein isoforms production or mRNA stability, contributing to transcriptome and proteome diversity. Almost 95% of human genes with multiple exons undergo alternative splicing events with a frequency higher than 10%, underscoring the pivotal roles of alternative splicing in cellular pathophysiology [4, 5]. In fact, alternative splicing has been demonstrated to play roles in plenty of key biological processes and human diseases, including several cancers. Mutations in cis-acting splicing elements and alterations of several splicing factors can dramatically change the splicing patterns of cancer-involved genes, contributing to tumorigenesis and cancer progression [6, 7]. Recent technological progress in RNA sequencing has provided enormous data for genome-wide analysis of alternative splicing patterns in cancers, for example, genome-wide analysis of differentially expressed splicing isoforms in ccRCC were conducted with Affymetrix Exon Array platform [8]. Furthermore, our previous study identified that splicing factor SF3B3 regulated the alternative splicing of EZH2 exon 14, and SF3B3 expression and splicing pattern of EZH2 might possess prognostic and therapeutic potential [9]. These studies imply that specific alternative splicing pattern may remarkably contribute to more reliable definition of molecular biomarkers for cancer early diagnosis and prognosis, and may translate into effective therapeutic targets. However, there is only a sparse body of research that investigates the aberrant splicing events and underlying splicing mechanisms in ccRCC.

In this study, we systematically identified the alternative splicing events with bioinformatic methods using RNA-sequencing data from The Cancer Genome Atlas (TCGA), and selected a series of significantly dysregulated splicing events including coiled-coil domain containing 50 (CCDC50) in ccRCC for further validation. CCDC50 was firstly characterized as chromosome 3 open reading frame 6 and mapped to chromosome 3q28, subsequent genome sequencing of CCDC50 validated its involvement in autosomal dominant nonsyndromic hearing loss [10, 11] while denied its causative effect for spastic paraplegia [12]. The truncated variant of CCDC50, has been identified as a tyrosine - phosphorylated and ubiquitinated protein. Upon epidermal growth factor (EGF) stimulation, the truncated CCDC50 protein could be phosphorylated at tyrosine 145 and 146, and then functioned as an inhibitor for the ligand - induced downregulation of epidermal growth factor receptor (EGFR) [13]. Furthermore, the truncated CCDC50 was proved to be phosphorylated on tyrosine residues by Src family kinases, acting as a negative regulator for the nuclear factor-kappa B (NF-κB) - mediated apoptotic pathway [14, 15]. However, CCDC50 is not fully studied in cancer contexts. One research project revealed that CCDC50 might be dispensable for cell survival in mantle cell lymphoma and chronic lymphocytic leukemia [16]. CCDC50 gene is comprised of 12 exons and the inclusion or skipping of exon 6 can generate full-length or short transcript, respectively. These two mRNA have differential expression levels in different human tissues, while the predominant transcript is the shorter one [12]. In addition, an article published recently suggested that CCDC50 short transcript might serve as a diagnostic and prognostic biomarker and probably a promising therapeutic target in hepatocellular carcinoma [17]. Nevertheless, no researchers have elaborated the specific pathophysiological functions of CCDC50 or the clinical significance and regulatory mechanism of CCDC50 pre-mRNA splicing in the context of ccRCC thus far.

In this study, we firstly validated the bioinformatic result of aberrant CCDC50 splicing in our renal cancer samples. Then we evaluated the clinical significance of splicing patterns of CCDC50 in survival prediction, and examined the distinct biological functions of different CCDC50 isoforms in ccRCC with a series of in vitro and in vivo experiments. Furthermore, we sought out the splicing regulatory mechanism of CCDC50 splicing, and identified the oncogenic splicing factor heterogeneous nuclear ribonucleoprotein A1 (HnRNP A1) was involved in the regulation of exon 6 inclusion/skipping in ccRCC. In addition, the oncogenic transcriptional factor zinc finger protein 395 (ZNF395) seemed to serve as a downstream molecule of shorter isoform of CCDC50. Overall, our findings suggested that HnRNP A1 - regulated aberrant alternative splicing of CCDC50 could contribute to the carcinogenesis and progression of ccRCC by modulating ZNF395.

## Methods

### Patient samples and clinical information

Forty-eight pairs of ccRCC samples and corresponding adjacent noncancerous tissues were obtained from primary ccRCC patients who underwent radical or partial nephrectomy in Tongji hospital between January 2015 and December 2017. The usage of human specimens was approved by the ethics committee of Tongji medical college, Huazhong University of Science and Technology, and written informed consent was obtained from each patient before surgery. The medical records of these patients were retrieved, and demographic characteristics, clinicopathological information, and survival data were recorded and analyzed in our further study.

### Cell lines and cell culture

Human renal cancer cell lines (786-O, A498, OS-RC-2) were cultured in RPMI-1640 medium containing 10% fetal bovine serum (FBS) at 37 °C in humidified atmosphere with 5% CO_2_, while other renal cancer cell line (ACHN), normal renal epithelial cells human kidney 2 (HK-2), and human embryonic kidney 293 (HEK293) were maintained in DMEM with 10% FBS.

### Plasmids and stable transfected cells establishment

Target fragments were inserted into lentiviral vectors such as pCDH-MSCV-MCS-EF1-copGFP (System biosciences, USA) and pSiCOR (Addgene, #11597), all plasmids were verified by DNA sequencing. Together with pGC-LV, pHelper 1.0, and pHelper 2.0 plasmids, recombinant lentiviral vectors were transfected into HEK293 cells, in which recombinant lentivirus was generated. Target cells were infected with lentivirus, then treated with puromycin for 14 days. After the efficiency of overexpression or depletion plasmids was confirmed, surviving cells were used for further experiments.

### RNA preparation and PCR

Total RNAs of cells or tissues were extracted using TRIzol reagent (Invitrogen, USA), and then reverse transcribed into cDNA using the Prime-Script™ one step real-time polymerase chain reaction (RT-PCR) kit (TAKARA, China). Semi-quantitative RT-PCR was performed with 2× Taq PCR Master Mix (Thermo Fisher Scientific, USA). GAPDH was used as internal control. RT-qPCR was performed using SYBR Green Mix (Roche, Germany). All primers used in our study were listed in Supplementary table 1 (Additional file 1).

### Fluorescence in situ hybridization (FISH)

FISH was performed on 12 pairs ccRCC and corresponding normal tissues in Wuhan Servicebio Technology following the manufacturer’s protocol. We labelled the truncated or full-length transcript with green or red fluorescence, respectively. The probe for truncated transcript was located at the junction fragment of exon 5 and exon 7, while probe for full-length transcript at exon 6. The fluorescence dots were counted by two experienced pathologists to represent the RNA expression of two CCDC50 isoforms.

### Colony formation, EdU incorporation, and MTS assay

In colony formation assays, approximately 1000 cells were seeded into six-well plates and cultured for two-weeks, the numbers of cell colonies were calculated after staining cells with crystal violet. In EdU incorporation assays, nucleus of proliferative cells were stained with red fluorescence while all nucleus could be stained with blue fluorescent light. In MTS assay, cells were treated with corresponding kit and then seeded into 96-well microplates at a density of 1000 cells per well, and the absorbance at 490 nm of each well was measured at different time points.

### Transwell assay

About 1 × 10^5^ of 786-O cells or 1.5 × 10^5^ OS-RC-2 cells were plated in the upper chambers of 24-well Transwell plates (Corning, USA) in FBS-free medium, and complete medium with 10% FBS was deposited in the lower chambers to serve as a chemo-attractant. For in vitro migration assay, cells which passed through the Transwell filter after 12 h were remained and stained by crystal violet. For in vitro invasion assay, Transwell membranes were coated with Matrigel prior to plating cells, cells which passed through the Matrigel membrane and Transwell filter after 24 h were stained and calculated. The relative number of passed cells represented the cells’ abilities of migration or invasion.

### Antibodies

Following antibodies were used in western blot: anti-CCDC50 (ab127169, Abcam), anti-ZNF395 (11759–1-AP, Proteintech), anti-HnRNP A1 (ab5832, Abcam), anti-β-actin (BM0627, Boster), anti-PCNA (10205–2-AP, Proteintech), anti-Cyclin D1 (60186–1-Ig, Proteintech), N-Cadherin (22018–1-AP, Proteintech), anti-Vimentin (BM0135, Boster), anti-ZEB1 (3396, Cell Signaling Technology), anti-VEGF (19003–1-AP, Proteintech), goat anti-mouse IgG HRP-linked whole antibody (31,430, Thermo Scientific), and goat anti-rabbit secondary antibody (31,460, Thermo Scientific).

### RNA immunoprecipitation (RIP)

RIP experiments were implemented to analyze the binding of HnRNP A1 to CCDC50 mRNA using Magna RIP Kit (17–701, Millipore) according to the manufacturer’s instructions.

### Animal experiments and metastasis assay

For the subcutaneous injection experiment, 5 × 10^6^ OS-RC-2 cells were injected subcutaneously into 8 mice per group at a single site. Tumor sizes were measured and calculated every 5 days. At day 25, mice were executed and tumors were excised and weighted. For the caudal vein injection experiment, 1 × 10^6^ OS-RC-2 cells were injected into 4 mice per group at the tail vein. Finally, lungs were resected and prepared for hematoxylin and eosin (H.E.) staining.

### Statistical analysis

The data were presented as the mean ± standard deviation (SD). Differences among groups were determined by a two-way analysis of variance followed by a post hoc Tukey test. Comparisons between two groups were performed using an unpaired Student t test. Survival curve was plotted using the Kaplan-Meier method and compared with the log-rank test. A value of *P* < 0.05 was considered as statistically significant. *P* < 0.05, *P* < 0.01 and *P* < 0.001 were marked as ‘*’, ‘**’, ‘***’.

## Results

### Bioinformatic analysis identify dysregulated CCDC50 exon 6 splicing in KIRC

The dysregulation of alternative RNA splicing plays a critical role in tumor development and progression. However, the roles of spliced variants and splicing factors that control splicing dysregulation in ccRCC carcinogenesis are still largely unexplored. In order to have a better understanding of the splicing events in ccRCC, we firstly analyzed the RNA-seq data of TCGA. We obtained the exon skip data of Kidney renal clear cell carcinoma (KIRC) from TCGA SpliceSeq Database (http://bioinformatics.mdanderson.org/TCGASpliceSeq/singlegene.jsp). This database provided the splicing information of 533 tumor samples and 72 normal tissues, so the data of 72 pairs of ccRCC tissues and corresponding adjacent noncancerous tissues were analyzed. The mean percent spliced-in index (PSI) value in both tumor samples and paired normal tissues were calculated and statistically compared. Candidate exon skip events in ccRCC were identified if the absolute difference value between cancer group and normal group was higher than 0.3 with statistical significance (Fig. 1a).

**Fig. 1:** CCDC50 exon 6 skipping event is significant in ccRCC and is correlated to poor prognosis. **a** Flow chart of the screening process of CCDC50 alternative splicing event. The data of 72 pairs of ccRCC and adjacent noncancerous tissues in TCGA were analyzed. The percent spliced-in (PSI) value were calculated and candidate exon skipping events were identified when the absolute difference value between the cancer group and normal one was higher than 0.3 with statistical significance. **b** The PSI value of CCDC50 exon 6 in 72 pairs of ccRCC and adjacent noncancerous tissues was calculated. **c** The PSI values of CCDC50 exon 6 in 33 types of cancer and normal tissues were acquired from TCGA SpliceSeq Database. Significantly lower mean PSI in tumor tissues was showed in KIRC. **d** The relative expression level of CCDC50 exons in ccRCC and normal tissues. **e** Kaplan-Meier curve showing (a) recurrence free survival and (b) overall survival of renal cancer patients in TCGA with high or low PSI values of CCDC50. (P_a_ = 0.0212, P_b_ = 0.5753 by log-rank test). **f** Kaplan-Meier curve showing (a) recurrence free survival and (b) overall survival of 48 ccRCC patients from Tongji Hospital with high or low PSI values of CCDC50. (P_a_ = 0.0240, P_b_ = 0.0469 by log-rank test)

Dysregulated CCDC50 exon splicing was identified as a candidate splicing event after our analysis. The mean PSI in 72 tumors and all 533 tumors was 0.081 ± 0.049 and 0.124 ± 0.142, while the mean PSI in 72 paired normal tissues was 0.468 ± 0.146 (*p* < 0.01) (Fig. 1b). Apart from KIRC, significantly lower mean PSI in tumor tissues was also found in many types of other cancer (Fig. 1c). Furthermore, we retrieved the relative expression data of each exon of CCDC50 in ccRCC samples, which showed that the expression levels of all exons were significantly higher in renal cancer except for exon 6, with an attenuated expression in tumor tissues (Fig. 1d). We further evaluated the significance of CCDC50 alternative splicing for prognosis prediction using TCGA data. Kaplan-Meier curves showed that higher PSI was associated with better recurrence-free survival (hazard ratio [HR]: 0.6425, 95% confidence interval [CI]: 0.4421–0.9337, *p* = 0.0212) (Fig. 1Ea), although higher PSI had no significant predictive value for overall survival (HR: 0.9167, 95% CI: 0.6762–1;243, *p* = 0.5753) (Fig. 1Eb). Moreover, we investigated the relationship of CCDC50 alternative splicing and prognosis of 48 patients from our hospital. Interestingly, Kaplan-Meier curves showed that higher PSI was significantly related to both better recurrence-free survival (HR: 0.3901, 95% CI: 0.1573–0.9674, *p* = 0.0240) (Fig. 1Fa) and overall survival (HR: 0.3593, 95% CI: 0.1288–1.002, *p* = 0.0469) (Fig. 1Fb).

### Alternative splicing of CCDC50 is aberrant in renal cancer tissues, cell lines, and is related to poor clinicopathological features

The CCDC50 gene can generate two mRNA transcripts through pre-mRNA alternative splicing. The pre-mRNA of CCDC50 consists of 12 exons and 11 introns. Exon 6 (528 bp) can be regulated by alternative splicing, and skipping and inclusion of exon 6 can generate the truncated (CCDC50-S) or full-length transcript (CCDC50-FL), respectively. The length of coding sequence (CDS) for different transcript is 921 bp and 1449 bp, which further generates protein products with 306 or 482 amino acids (Fig. 2a). We made further efforts to explore whether the expression pattern of CCDC50 transcripts existed in our ccRCC and normal tissues or renal cell lines. Semi-quantitative RT-PCR analysis of 12 pairs of ccRCC samples and corresponding noncancerous tissues revealed that CCDC50-FL was predominately examined in normal tissues and barely appeared in ccRCC tissues, while CCDC50-S was significantly more abundant in cancerous tissues (Fig. 2b). Moreover, compared to human immortalized kidney proximal tubular cell HK-2, all renal cancer cell lines showed notable elevated expression of CCDC50-S, while the full-length transcript was quenched in cancer cells (Fig. 2c). We also examined the subcellular localization of CCDC50 protein isoforms, both isoforms localized in the cytoplasm of OS-RC-2 cells (Fig. 2d). Furthermore, we conducted RT-qPCR using primers which amplified shared exons of both transcripts or separated exon 6 of CCDC50 to examine the expression of total CCDC50 transcripts and CCDC50-FL in 12 pairs tissues. The results demonstrated higher overall CCDC50 expression in majority of tumor samples, while exon 6 expression levels were significantly more abundant in normal tissues (Additional file 2, Supplementary Figure 1A-1B).

**Fig. 2:** CCDC50-S is upregulated in ccRCC tissues, cell lines, and is associated with poor clinicopathological features. **a** Schematic representation of CCDC50 pre-mRNA and two alternatively spliced mRNA isoforms. Exon 6 (528 bp) is spliced-out in CCDC50-S and spliced-in in CCDC50-FL. **b** Expression of CCDC50-S and CCDC50-FL mRNA in 12 pairs ccRCC (T) and adjacent noncancerous tissues (N) by RT-PCR. GAPDH was used as the internal control. **c** Expression of CCDC50-S and CCDC50-FL mRNA in normal human kidney 2 (HK2) cell line and four renal cancer cell lines (ACHN, OS-RC-2, 786-O, A498) by RT-PCR. GAPDH was used as the internal control. **d** Subcellular localization of CCDC50 protein isoforms in OS-RC-2 cells. Blue fluorescence for DAPI and red fluorescence for CCDC50 isoforms. **e** The expression of CCDC50-S and CCDC50-FL in 12 pairs ccRCC and normal tissues was determined by Fluorescence in Situ Hybridization (FISH). Representative images of 2 pairs tissues are shown. Blue fluorescence for DAPI, green fluorescence for CCDC50-S and red fluorescence for CCDC50-FL. **f** The association between CCDC50 isoforms mRNA expression and (a) tissue types, (b) ccRCC T stage and (c) ccRCC Fuhrman Grade were analyzed. Quantitative data are presented as the mean ± SD

To further validate the aberrant alternative splicing of CCDC50, we conducted FISH to label CCDC50-S with green fluorescence and CCDC50-FL with red fluorescence using 12 pairs ccRCC and corresponding normal tissues. The results showed that CCDC50-S was extremely elevated in tumor samples, while paired normal samples presented significantly more CCDC50-FL, which is in accordance with the results above (Fig. 2E-Fa). We next assessed the association between the expression of CCDC50 transcripts and clinicopathological features. We found that CCDC50-S expression increased significantly when T stage and Fuhrman Grade advanced, although CCDC50-FL showed no significant difference (Fig. 2Fb-Fc).

### Diverse splicing variants exert opposite tumorigenic effects in vitro and in vivo

We first assessed the tumorigenic effects of CCDC50 isoforms on ccRCC cells to have a better understanding of the importance of CCDC50 in regulating renal cancer biology. RCC cell lines stably overexpressing CCDC50-S or CCDC50-FL, and stably silencing the CCDC50 transcripts with short hairpin RNA (shRNAs) were constructed and validated (Additional file 2, Supplementary Figure 2A-2B). Stable overexpression of CCDC50-S in RCC cell lines accelerated the cell proliferation and survival abilities as shown by colony formation, EdU incorporation assay and MTS, while ectopic expression of CCDC50-FL exhibited opposite effects on cells (Fig. 3a-c). Besides, two shRNAs which deprived the mRNA and protein expression of CCDC50 significantly repressed the cell proliferation (Fig. 3a-c). We also performed Transwell assays to examine the cell migration and invasion abilities, the results showed that CCDC50-S overexpression significantly promoted cell migration and invasion, but CCDC50-FL exerted adverse effects (Fig. 3d-e). Furthermore, the silence of CCDC50 transcripts obviously inhibited cell migration and invasion (Fig. 3d-e). Given that the predominant transcript of CCDC50-S, these results validated that CCDC50-S exerted an oncogenic function on ccRCC in vitro*,* while CCDC50-FL played tumor-suppressive roles in ccRCC.

**Fig. 3:** CCDC50-S and CCDC50-FL exert opposite tumorigenic effects in vitro and in vivo. **a** Colony formation assays were conducted in 786-O and OS-RC-2 cells with CCDC50-S/CCDC50-FL overexpression or CCDC50 silence. The presented data are means ± SD in three independent experiments. **b** EdU incorporation assays were performed in CCDC50-S/CCDC50-FL overexpressed or CCDC50 silenced 786-O and OS-RC-2 cells. The percent of proliferating cells (Red fluorescence) in total cells (blue fluorescence) was calculated. **c** 786-O and OS-RC-2 cells expressing CCDC50-S/CCDC50-FL or sh-CCDC50 were implemented with MTS assays to assess cell viability. **d-e** The migration and invasion ability of CCDC50-S/CCDC50-FL or sh-CCDC50 stably transfected 786-O and OS-RC-2 cells was determined by Transwell assays. **f** OS-RC-2 cells expressing CCDC50-S/CCDC50-FL or sh-CCDC50 and corresponding control plasmids were injected subcutaneously into mice. Isolated tumors were presented and their volume and weight were calculated. **g-h** CCDC50-S/CCDC50-FL overexpressed or CCDC50 silenced OS-RC-2 cells were injected subcutaneously into mice caudal vein. The lung metastasis imaging and H.E. staining images were presented. Red arrows meant lung metastases

Xenograft experiments in immunodeficient mice also supported this conclusion, as OS-RC-2 cells with CCDC50-S overexpression exhibited accelerated tumor growth velocity and larger tumors, while CCDC50-FL in OS-RC-2 cells emerged as inhibitor for tumor growth (Fig. 3f). Additionally, OS-RC-2 cells with sh-CCDC50 inhibited tumor growth significantly (Fig. 3f). Furthermore, we constructed caudal vein injection model and performed H.E. staining on lung metastases in order to assess the metastasis ability of OS-RC-2 cells with different transcripts. The results validated that CCDC50-S promote tumor metastasis, but CCDC50-FL and sh-CCDC50 suppressed tumor metastasis ability (Fig. 3g-h).

### HnRNP A1 promotes the skipping of exon 6 of CCDC50 pre-mRNA

Alternative splicing is strictly regulated by the interaction between multiple trans-acting proteins and corresponding cis-acting silencers and enhancers on the pre-mRNA [18]. Splicing factors are regulatory proteins with pre-mRNA - binding potential, such as serine and arginine-rich (SR) proteins and heterogeneous nuclear ribonucleoproteins (hnRNPs). Firstly, using TCGA gene expression RNAseq data, we sought to identify splicing factors with differential expression in ccRCC (data not shown). Besides, we previously found that many splicing factors presented differential expression in renal cancer by microarray [19]. We reasonably conjectured that among these differentially expressed splicing factors, some might regulate the CCDC50 alternative splicing. Thus, in order to explore the effects of splicing factors on CCDC50 pre-mRNA splicing, we constructed a series of shRNA plasmids targeting these splicing factors, namely HnRNP A1, HnRNP A2B1, HnRNP A3, HnRNP H3, PTBP1 (HnRNP I), PSIP1, SFPQ, SRPK3, SRSF1, SF3A1, SF3A2, SF3B3. Furthermore, we constructed overexpression plasmids of several splicing factors according to our initial semi-quantitative RT-PCR results. We then treated HEK293 cells with these plasmids of interest and control plasmids, and examined the expression of two isoforms via semi-quantitative RT-PCR. Combining the TCGA expression data with our PCR results, we found that HnRNP A1 promoted the skipping of exon 6, which was proved by the increase of the PSI (portion of full-length transcript) by sh-HnRNP A1 and obvious decrease of PSI by HnRNP A1 overexpression (Fig. 4a). Furthermore, Pearson correlation analysis indicated that the relative expression of HnRNP A1 was negatively correlated with the expression level of CCDC50 exon 6 (*r* = − 0.361, *p* < 0.0001) in TCGA cohort (Fig. 4b), which was in accordance with the theory that HnRNP A1 impeded the inclusion of exon 6 and decreased the proportion of full-length transcript. As we have shown in Fig. 2c, we did not detect any full-length CCDC50 transcript in RCC cell lines, therefore, we had to construct a splicing minigene which included the full-sequence of exon 5, exon 6, exon 7 and flanking part of intron 5 and intron 6. This minigene generated two transcripts with length of 722 bp and 198 bp (Fig. 4c). After stably transfecting 786-O and OS-RC-2 cells with minigene, we treated these cells with HnRNP A1 expressing vector or shRNAs against HnRNP A1. The results in 786-O (Fig. 4Da) and OS-RC-2 (Fig. 4Db) both demonstrated that HnRNP A1 overexpression decreased the full-length transcript while knockdown of HnRNP A1 increased the relative expression of full-length transcript. Furthermore, we examined the regulation effect of HnRNP A1 on CCDC50 at protein level in cells transfected with HnRNP A1 or sh-HnRNP A1 plasmids, and the results confirmed the conclusion of minigene experiment (Fig. 4Ea-Eb). In addition, using the RIP with anti-HnRNP A1 antibody, we detected an enrichment of CCDC50-S and pre-mRNA sequence on HnRNP A1 protein, which validated that HnRNP A1 could bind to CCDC50 pre-mRNA (Fig. 4f). These data also strengthened our conclusion that HnRNP A1 could regulate the alternative splicing of CCDC50 pre-mRNA by promoting skipping of its exon 6.

**Fig. 4:** HnRNP A1 promotes the skipping of exon 6 and exclusion of CCDC50 pre-mRNA. **a** CCDC50 splicing regulator was screened from a series of splicing factors using RT-PCR in HEK293 cells. GAPDH was used as the internal control. **b** Negative correlation between the expression level of CCDC50 exon 6 and HnRNP A1 was observed in ccRCC samples (*r* = − 0.361, *p* < 0.0001). **c** Minigene including the full sequence of exon 5, exon 6, exon 7 and flanking part of intron 5 and intron 6 was designed and constructed. **d** Regulation role of HnRNP A1 on CCDC50 splicing was validated by RT-PCR in (a) 786-O and (b) OS-RC-2 cells, after the minigene and HnRNP A1 or sh-HnRNP A1 plasmid were transfected. GAPDH was used as the internal control. **e** Regulation role of HnRNP A1 on CCDC50 splicing was comfirmed by western blot in (a) 786-O and (b) OS-RC-2 cells, after the HnRNP A1 or sh-HnRNP A1 plasmid were transfected. β-actin was used as the internal control. **f** Binding of HnRNP A1 with CCDC50-S and pre-mRNA sequences was confirmed by RNA immunoprecipitation (RIP) in 786-O cells

### HnRNP A1 functions as an oncogenic splicing factor in ccRCC

Since the role of HnRNP A1 in renal cancer remain undiscovered, we further explored its expression level and biological functions in ccRCC. TCGA data showed that HnRNP A1 was significantly overexpressed in KIRC (Additional file 2, Supplementary Figure 3A). Then, we evaluated the expression pattern of HnRNP A1 in renal cancer cell lines, which validated the overexpressed pattern of HnRNP A1 in these cell lines (Additional file 2, Supplementary Figure 3B). Together, these revealed that HnRNP A1 expression level might help to predict the prognosis of ccRCC patients.

In addition, we studied the biological functions of HnRNP A1 in renal cancer cell lines. We constructed and validated renal cancer cell lines stably overexpressing HnRNP A1 and stably silencing HnRNP A1 with shRNA (Additional file 2, Supplementary Figure 4). As shown in Fig. 5a-c, knockdown of HnRNP A1 significantly reduced the proliferative ability of 786-O and OS-RC-2 cells, while ectopic expression of HnRNP A1 increased these capacities of renal cancer cells. Moreover, Transwell assay supported that HnRNP A1 could increase the migration and invasion capacities of two renal cancer cell lines (Fig. 5d-e).

**Fig. 5:** HnRNP A1 is an oncogene in ccRCC. **a** The proliferative ability was assessed by colony formation assays in 786-O and OS-RC-2 cells expressing HnRNP A1 or sh-HnRNP A1. **b** EdU incorporation assays were conducted to acquire the percent of proliferating cells in HnRNP A1 overexpressed or sh-HnRNP A1 silenced 786-O and OS-RC-2 cells. **c** The cell viability was determined by MTS assays in 786-O and OS-RC-2 cells expressing HnRNP A1 or sh-HnRNP A1. **d-e** 786-O and OS-RC-2 cells with HnRNP A1 overexpression or HnRNP A1 knockdown were subjected to Transwell migration and invasion assay

We further conducted rescue assay to evaluate the regulatory correlation between CCDC50 and HnRNP A1. Overexpression of CCDC50-S could reverse the reduction of proliferation and migration ability caused by HnRNP A1, while overexpression of CCDC50-FL had no significant effect (Additional file 2, Supplementary Figure 5A-5C). These findings consolidated our theory that HnRNP A1 could exert its oncogenic function in ccRCC through modulating the alternative splicing of CCDC50 and increasing the relative expression of truncated CCDC50.

### ZNF395 is a downstream oncogenic factor of CCDC50-S

As the truncated transcript of CCDC50 was the predominant transcript which exerted oncogenic functions, we sought to identify its downstream molecules and corresponding mechanism which explained its roles in ccRCC. Through digging from TCGA data and the RNAseq data from previous article about CCDC50, we found that ZNF395, PFKFB4, SLC2A3, LAMP1, BNIP3L and TP53I3 were among the most affected proteins after CCDC50 knockdown. Because CCDC50-S was the main transcript and CCDC50-FL was hard to detect in renal cancer tissues and cell lines, we used CCDC50 knockdown plasmid to represent the knockdown of CCDC50-S. Our RT-qPCR and western blot results validated that the mRNA and protein expression levels of ZNF395 were attenuated after CCDC50 knockdown in vitro, and the tendency was reversed after ectopic expression of CCDC50-S (Fig. 6Aa and Ab), while the other candidate genes were not obviously influenced by CCDC50 knockdown or overexpression (data not shown). Interestingly, RT-qPCR also showed that CCDC50-FL overexpression could attenuate the expression level of ZNF395 (Additional file 2, Supplementary Figure 6). Furthermore, our RT-qPCR results in renal cancer cell lines and 12 pairs ccRCC tissues elucidated the enhanced expression pattern of ZNF395 (Fig. 6Ba and Bb). Kaplan-Meier curve also indicated that higher expression of ZNF395 was significantly capable of predicting worse overall survival of ccRCC patients in TCGA (Additional file 2, Supplementary Figure 7). RNA-seq data in 17 cancer types generated by the TCGA demonstrated the enriched expression of ZNF395 in renal cancer compared to other cancer types (Additional file 2, Supplementary Figure 8), which highlighted the possible pivotal roles of ZNF395 in ccRCC carcinogenesis.

**Fig. 6:** ZNF395 is a downstream oncogene of CCDC50-V1. **a** The expression of ZNF395 was determined in 786-O and OS-RC-2 cells by (a) RT-qPCR and (b) western blot after the CCDC50 knockdown or CCDC50-S overexpression. GAPDH and β-actin were used as the internal control of RT-qPCR and western blot respectively. **b** The expression of ZNF395 was examined in (a) normal HK2 cell line and four renal cancer cell lines (ACHN, OS-RC-2, 786-O, A498), (b) ccRCC and corresponding normal tissues by RT-qPCR. GAPDH was used as the internal control. **c** Colony formation assays were utilized to examine the proliferative ability of 786-O and OS-RC-2 cells with ZNF395 knockdown. **d** EdU incorporation assays were conducted in ZNF395 silenced 786-O and OS-RC-2 cells. **e-f** Migration and invasion assay were performed in 786-O and OS-RC-2 cells expressing sh-ZNF395. **g** Western blot was implemented to identify downstream genes and pathways of ZNF395 in 786-O and OS-RC-2 cells. β-actin was used as the internal control

After the RCC cell lines stably overexpressing ZNF395 or silencing ZNF395 with shRNA was constructed and validated (Additional file 2, Supplementary Figure 9), we made an inquiry for the specific roles of ZNF395 in renal cancer. The colony formation, EdU, and Transwell assays proved unequivocal evidence that ZNF395 was a pro-proliferative protein which also promoted cell migration and invasion (Fig. 6c-f). We further conducted western blot to find that ZNF395 exerted its oncogenic function through proliferation, epithelial - mesenchymal transition (EMT), and angiogenesis pathways (Fig. 6g).

### High CCDC50-S / high HnRNP A1 is associated with poor overall survival

Finally, we evaluated the association of CCDC50-S combined with HnRNP A1 or ZNF395 and the overall survival of renal cancer patients in TCGA. Kaplan-Meier curves showed that high CCDC50-S / high HnRNP A1 was associated with poor overall survival (*p* = 0.0079), while there was no significant relation between high CCDC50-S / high ZNF395 and overall survival (*p* = 0.64) (Additional file 2, Supplementary Figure 10A-10B).

## Discussion

This study firstly sketched the aberrant exon skipping profiling in ccRCC with TCGA dataset, and proved the reliability of this profiling by validating the aberrant splicing of CCDC50 exon 6 in independent ccRCC cohort. We also observed that splicing factor HnRNP A1 could exert it carcinogenic functions in ccRCC via promoting the skipping of exon 6 of CCDC50 pre-mRNA and increasing the proportion of oncogenic truncated transcript of CCDC50. Besides, transcriptional factor ZNF395 could become a downstream effector of CCDC50 to regulate the carcinogenesis of ccRCC. Furthermore, the splicing pattern of CCDC50 and the expression level of HnRNP A1 and ZNF395 might have the potential to predict the prognosis of ccRCC patients. Our findings not only identified a common and important splicing event in ccRCC, but also provided integrated regulatory network which elucidated the mechanism of exon skipping involving in renal cancer progression.

CCDC50 had been studied in several cellular contexts and some human diseases, which indicated its vital involvement in epidermal growth factor - mediated cell signaling, NF-κB and Fas signaling pathways [14, 15, 20]. Additionally, mutation of CCDC50 gene or de novo deletion of 3q29 which compromised CCDC50 gene was shown to cause progressive hearing loss in several studies [10, 11, 21], underlining the critical functions of CCDC50 in human.

However, there were only sparse studies which implied the involvement of CCDC50 in carcinogenesis or progression of human cancers. Farfsing et al. demonstrated that CCDC50 was required for the survival of mantle cell lymphoma and chronic lymphocytic leukemia cells through gene knockdown assays [16]. Chuang et al. identified that copy number gain of CCDC50 was more common in cyclin D1-negative pleomorphic mantle cell lymphoma, but the significance of this finding was still elusive [22]. Wang et al. demonstrated that serine- and arginine-rich splicing factor 3 (SRSF3) could directly bind to CCDC50-S mRNA to maintain its stability in the cytoplasm, which enhanced oncogenic progression of hepatocellular carcinoma through the Ras/Foxo4 signaling pathway [17]. Although they revealed the oncogenic role of CCDC50-S, the function of CCDC50-FL was not analyzed [17]. Besides, the mechanism that Wang et al. uncovered between SRSF3 and CCDC50-S was molecule stability regulation rather than alternative splicing regulation [17]. Interestingly, Wang et al. also found that the BaseScope signal of CCDC50-S mRNA was relatively negative in eight types of solid tumors including renal cancer [17], but we validated the existence of CCDC50-S in ccRCC and further investigated its biological function.

Currently, the expression pattern, biological functions and underlying molecular mechanisms of CCDC50 in ccRCC remain poorly defined. We found that CCDC50 was upregulated in ccRCC and the predominant CCDC50 transcript exerted an oncogenic function in ccRCC, which was consistent with the pro-survival function shown by Fartsing et al. [16]. Like the majority of human genes, CCDC50 locus could generate diverse mRNA transcripts through the alternative splicing of pre-mRNA. Tashiro et al. noticed that two splice variants of CCDC50 were ubiquitously expressed in human tissues and the short one is dominantly expressed, they also found that long isoform of CCDC50 protein had significantly lower affinity for binding to EGFR [13]. However, they failed to identify the distinct functions of CCDC50 isoforms, let alone the human cancer contexts. Our results were conformed with previous findings, and we further elucidated that dysregulation of alternative splicing of CCDC50 was a normal phenomenon in ccRCC. Furthermore, we provided reliable evidence that truncated or full-length CCDC50 could promote or inhibit the proliferation, migration, invasion, and tumor growth of renal cancer, respectively. The relative expression of tumor-suppressive CCDC50-FL was diminished in ccRCC, while the concentration of oncogenic CCDC50-S significantly increased in this malignancy. An increasing body of literature shows that dysregulation of pre-mRNA splicing contributes to tumorigenesis and turns into potent drivers of malignant phenotypes [6, 23], our results indicated that CCDC50 could also be regarded as an outstanding example because the splicing pattern of CCDC50 could predict survival of ccRCC patients. Notably, some compounds have been developed to affect splicing control and have resulted in promising therapeutic agents [24], thus developing novel anticancer compounds targeting alternative splicing of CCDC50 might become eligible strategy for controlling cancers including ccRCC.

HnRNPs are a set of ~ 20 abundant proteins which involve in several post-translational modifications such as splicing of introns, 5′-end capping, and polyadenylation [25]. HnRNP A1 is the most abundant and ubiquitously expressed HnRNPs which can shuttle between the nucleus and cytoplasm via its Gly-rich auxiliary domain [26], which endows it with more convenience to regulate RNA maturation and pre-mRNA splicing. HnRNP A1 has been demonstrated to be involved in several pathophysiological processes which drive the carcinogenesis and progression of many types of malignancies [27]. HnRNP A1 mainly plays oncogenic roles in the majority of cancer types, such as colon cancer [28] and hepatocellular carcinoma [29], while its functions in ccRCC are still elusive. HnRNP A1 is capable of preventing exon skipping of multiple genes [30]. For example, HnRNP A1 could bind to sequences flanking pyruvate kinase exon 9 and cause the exon 10 inclusion, increasing the PKM2/PKM1 ratio and promoting aerobic glycolysis in brain tumors [31, 32]. Current study found that HnRNP A1 was upregulated and exerted pro-tumorigenic functions in ccRCC, it could also regulate the alternative splicing of CCDC50 to promote truncated CCDC50 transcript production. These data shed light on how splicing factor HnRNP A1 contributed to the tumor progression. However, more thorough inquiry into the binding site of HnRNP A1/CCDC50 pre-mRNA and specific molecular mechanisms of splicing regulation was still imperative.

ZNF395 was firstly identified as a papillomavirus binding factor which bound to SAP30 and negatively regulated gene transcription [33]. Additionally, ZNF395 could function as a transcriptional activator of several interferon-stimulated genes, such as CXCL10 and CXCL11 [34]. Further study indicated that ZNF395 could exert its transcriptional activation for proinflammatory factors and contribute to inflammatory microenvironment under HIF-1α dependent hypoxic conditions [35]. Moreover, Yao et al. proved that VHL deficiency in ccRCC drove enhancer activation of ZNF395, a ccRCC master regulator. VHL inactivation stabilized HIF-2α - HIF-1β heterodimer binding at the enhancers, and further activated the transcription of ZNF395 by recruiting histone acetyltransferase p300 on ZNF395 promoter [36]. In our study, we found that ZNF395 was a downstream protein of CCDC50, which was consistent with the genome-wide expression profile after CCDC50 modulation [16]. Short CCDC50 isoform could suppress the degradation and internalization of EGF receptor on plasma membrane [13], resulting in the accumulation of active EGFR on plasma membrane. EGFR stimulation could induce the downstream AKT activation, leading to the phosphorylation and subsequent activation of p300 [37]. Activated p300 continued to increase the transcriptional activity of ZNF395, explaining the upregulation of ZNF395 after treating with short CCDC50 isoform. Besides, HIF-2α accumulation under hypoxic microenvironment could promote EGFR mRNA translation and diminish the necessity for EGFR mutations [38], the mutual promotion of EGFR and HIF-2α - p300 - ZNF395 pathway turned out to be significant driver of tumorigenic progression of ccRCC. On the other hand, we demonstrated that ZNF395 played its oncogenic role through proliferation, EMT, and angiogenesis pathways, which provided a comprehensive understanding of ZNF395 function in cancer.

The significance of CCDC50-S combined with HnRNP A1 or ZNF395 for prognosis prediction was revealed. High CCDC50-S / high HnRNP A1 could predicted poor overall survival, which was consistent with our conclusions. However, high CCDC50-S / high ZNF395 had no significant prognostic value. This might be explained by the small number of low CCDC50-S / low ZNF395 cases (only 44 cases). These results should be further validated by more studies with larger sample sizes.

## Conclusions

In summary, this study validates the aberrant splicing pattern of CCDC50 exon 6 initially identified by bioinformatic methods, and identifies oncogenic splicing factor HnRNP A1 as a regulator of CCDC50 exon 6 skipping in ccRCC. The predominant truncated transcript of CCDC50 promotes the tumorigenesis and progression of ccRCC via involving ZNF395 - related pathways, while full-length CCDC50 transcript plays tumor suppressive roles in malignancy transformation of ccRCC. Our findings provide complete exploration of CCDC50 exon 6 splicing, establishing novel therapeutic strategy for management of ccRCC. Besides, the splicing pattern of CCDC50, expression of HnRNP A1 and ZNF395 have potential prognostic value for ccRCC patients.

## Supplementary information

**Additional file 1.** Supplementary table 1. The primers used in the study.

**Additional file 2.** Supplementary figure 1–10.

## Data Availability

Not applicable.

## Abbreviations

ccRCC: clear cell renal cell carcinoma
CCDC50: Coiled-coil domain containing 50
pre-mRNA: precursor mRNA
CCDC50-FL: CCDC50 full-length transcript
CCDC50-S: CCDC50 truncated transcript
HnRNP A1: Heterogeneous nuclear ribonucleoprotein A1
ZNF395: Zinc finger protein 395
RCC: Renal cell carcinoma
VHL: Von Hippel-Lindau
HIFs: Hypoxia-inducible factors
TCGA: The Cancer Genome Atlas
EGF: Epidermal growth factor
EGFR: Epidermal growth factor receptor
NF-κB: Nuclear factor-kappa B
FBS: Fetal bovine serum
HK-2: Human kidney 2
HEK293: Human embryonic kidney 293
RT-PCR: Real-time polymerase chain reaction
FISH: Fluorescence in Situ Hybridization
RIP: RNA immunoprecipitation
H.E.: Hematoxylin and eosin
SD: Standard deviation
KIRC: Kidney renal clear cell carcinoma
PSI: Percent spliced-in index
HR: Hazard ratio
CI: Confidence interval
CDS: Coding sequence
shRNAs: short hairpin RNA
SR: Serine and arginine-rich
hnRNPs: heterogeneous nuclear ribonucleoproteins
EMT: Epithelial - mesenchymal transition
SRSF3: Serine- and arginine-rich splicing factor 3
